# Anti-Cancer Activities of Thyrointegrin α_v_β_3_ Antagonist Mono- and Bis-Triazole Tetraiodothyroacetic Acid Conjugated via Polyethylene Glycols in Glioblastoma

**DOI:** 10.3390/cancers13112780

**Published:** 2021-06-03

**Authors:** Kavitha Godugu, Mehdi Rajabi, Shaker A. Mousa

**Affiliations:** The Pharmaceutical Research Institute, Albany College of Pharmacy and Health Sciences, Rensselaer, NY 12208, USA; Kavitha.Godugu@acphs.edu (K.G.); m.rajabi.s@gmail.com (M.R.)

**Keywords:** anticancer, glioblastoma, anti-angiogenesis, thyrointegrin αvβ3, PEG, triazole tetrac, P-bi-TAT, P-m-TAT, tetrac

## Abstract

**Simple Summary:**

Different Triazole Tetrac (TAT) thyrointegrin αvβ3 antagonists exhibited optimal therapeutic efficacy against U87 or primary glioblastoma cells. TAT containing molecules bind with high affinity to the integrin αvβ3 and plasma protein Transthyretin (TTR), which facilitate transport across the blood brain barrier. Biological studies showed that decreasing the PEG linker size (1600 versus 4000) or having mono-TAT versus bi-TAT had no significant impact on their αvβ3 binding affinity, anti-angiogenesis, and overall anti-cancer efficacy.

**Abstract:**

Integrin αvβ3 receptors are overexpressed in different tumors and their associated neovascularization and hence, represent a potential cancer target. We previously synthesized a high affinity thyrointegrin αvβ3, P_4000_-bi-TAT (tetrac derivative), with potent anticancer properties. However, the long polydisperse PEG conjugate showed large scaleup and analytical/bioanalytical issues. Hence, in the present study, we synthesized a mono versus bi-triazole tetrac with discrete monodisperse PEG, which provided improvement in scaleup and bioanalysis. In the present study, we compared binding affinity and anticancer activates with a smaller PEG size (P_1600_-bi-TAT, Compound **2**) and the removal of one TAT molecule (P_1600_-m-TAT, Compound **3**) versus P_4000_-bi-TAT, Compound **1**. The results of the selectivity and affinity of TATs showed greater affinity to integrin αvβ3. The xenograft weights and tumor cell viabilities were decreased by >90% at all doses compared to the control (ON Treatment, *** *p* < 0.001) in cells treated with Compounds **1**, **2**, and **3** in U87-Luc-treated mice. The in vivo luminescent signals of U87-luc cells reflect the proliferation and distribution of tumor cells in the animals and the maximum intensity corresponding to the maximum tumor cells that the animals could tolerate. We found that the three thyrointegrin αvβ3 antagonists exhibited optimal therapeutic efficacy against U87 or primary glioblastoma cells. Biological studies showed that decreasing the PEG linker size (1600 vs. 4000) or having mono-TAT or bi-TAT had no significant impact on their αvβ3 binding affinity, anti-angiogenesis, or overall anti-cancer efficacy.

## 1. Introduction

Glioblastoma multiforme (GBM) is the most aggressive brain tumor with a high mortality rate [1,2]. Due to the severity of the disease, patients survive an average of only 12 months, and most do not survive beyond two years. Standard treatments of surgery, radiation, and conventional chemotherapy can increase the five-year survival rate to 5–8% [3,4]. Overall survival has been improved in clinical trial populations within the last few years from 12 months to 16 months. However, tumor heterogenicity and resistance mechanisms are expressed by GBM, which limits the effectiveness of therapeutic interventions.

Integrin αvβ3, a heterodimeric cell surface adhesion membrane receptor, is overexpressed in GBM at the tumor margins (invasive regions) and tumor-relevant blood vessels [5]. It has a high affinity for the protein components of the extracellular matrix (ECM) and plays an important role in cell invasion and motility, allowing for crosstalk between the cell and the surrounding stroma as well as with adjacent vascular growth factor receptors. The arginine–glycine–aspartate (RGD) recognition site on integrins αvβ3 is involved in ECM protein interactions and may activate signal transduction pathways. Thus, integrin αvβ3 plays a pleiotropic role in GBM, and the RGD domain is a therapeutic target for antitumor products, which has allowed for the development of various RGD-based antagonists, conjugates, and nanoparticles [6,7]. 

The extracellular domain of integrin αvβ3 bears a novel small molecule binding site that exclusively recognizes thyroid hormones and thyroid hormone analogs [8,9]. These analogs include tetraiodothyroacetic acid (tetrac), a deaminated derivative of I-thyroxine (T4), and a “thyrointegrin” antagonist that displaces I-triiodothyronine (T3) and T4 from the thyroid hormone analog receptor site on integrin αvβ3 and also initiates a number of intracellular actions via the integrin in the absence of T4 [9,10,11]. Our several previous studies showed that the nano-diamino-tetrac, (NDAT) based on poly(lactic-co-glycolic acid) (PLGA) that is conjugated to tetrac, have improved activity compared to tetrac alone at the integrin in terms of reduced cancer cell proliferation and induced apoptosis. These anticancer actions primarily reflect changes in the transcription of specific genes [12,13,14]. 

We recently synthesized a high affinity thyrointegrin αvβ3 antagonist, P-bi-TAT, a tetrac-based inhibitor with a triazole moiety on the outer ring of tetrac and covalently conjugated to a polymer via poly(ethylene glycol) (PEG, P) PEGylation (Compound **1**, Figure 1A). Thus, Compound **1** is a dimer, or bis triazole tetrac (TAT); P-bi-TAT has two tetrac molecules covalently bound via triazoles to PEG_4000_ (MW = 4000). It is effective against xenografts of human GBM. PEG modification affords a long-circulating property by evading macrophage-mediated uptake and removal from the systemic circulation. A PEG spacer allows the ligand to remain in the systemic circulation and provides flexibility to the attached ligand for efficient interaction with its target [11]. In spite of high binding to the αvβ3 receptor and favorable anticancer effects, these long polydisperse PEG conjugates of the molecule showed analysis issues in quality control and bioanalytical assays and also difficulty in its synthesis and scalability. Hence, in order to overcome these above issues, we synthesized a smaller PEG with a molecular weight of 1600 (Compound **2**, Figure 1B) and removed one TAT molecule of P-bi-TAT to form a mono-TAT agent, the P-m-TAT molecule (Compound **3**, Figure 1C), retaining the excellent solubility and potency of Compound **1**.

In this study, we tested the hypothesis that decreasing the PEG size from 4000 to 1600 MW and removing one TAT molecule of P-bi-TAT would improve its binding affinity and therapeutic value. An integrin αvβ3 binding assay was used to explore the binding modes of P_4000_-bi-TAT (Compound **1**), P_1600_-bi-TAT (Compound **2**), and P_1600_-m-TAT (Compound **3**), and we further evaluated their therapeutic efficacies using U87 glioma cells.

## 2. Materials and Methods

P_4000_-bi-TAT (Compound **1**), P_1600_-bi-TAT (Compound **2**), and P_1600_-m-TAT (Compound **3**) were synthesized in our laboratory according to our previously described method [11]. Dulbecco’s Modified Eagle Medium (DMEM), fetal bovine serum (FBS), penicillin, streptomycin, trypsin/EDTA, and bovine serum albumin (BSA) were purchased from Sigma-Aldrich (St. Louis, MO, USA). The human glioblastoma U87-luc cells U87-luc cells were from ATCC (Manassas, VA, USA), and the human primary GBM cells 052814, 021913, and 101,813 were a generous gift from the University at Pittsburgh Medical Center (Department of Neurosurgery). Purified αvβ3 and anti-αvβ3 conjugated with biotin were obtained from Bioss Inc. (Woburn, MA, USA), the streptavidin—HRP conjugates were from Thermo Fisher Scientific (Grand Island, NY, USA), the fibrinogen was from Millipore Sigma (Burlington, MA, USA), and the 3,3′,5,5′-tetramethylbbenzidine (TMB) and TMB-stop solution were from ABCAM Inc (Cambridge, MA, USA).

### 2.1. Binding Affinity of Compounds to Integrins Purified αvβ3 (1 µg/mL)

The binding affinity of Compounds **1**, **2**, and **3** to purified αvβ3 was measured using previously described methods with slight modifications [12,15,16,17]. Fibrinogen was coated to polystyrene microtiter plate wells and incubated at 4 °C overnight, and then the wells were blocked with 3% BSA for 2 h at room temperature. The wells were washed with Buffer A (50 mM Tris/HCl, 100 mM NaCl, 1 mM CaCl_2_, 1 mM MgCl_2_, 1% BSA) three times. Integrins αvβ1, αvβ3, αvβ5, αvβ6, IIbβ3, and α5β1 (ACRO Biosystems, Newark, DE, USA) and increasing concentrations of the compounds were added and incubated for 2 h at room temperature, and then the wells were washed three times with Buffer A and incubated with a streptavidin–HRP conjugate (1:1000 in Buffer A) for 1 h at room temperature. Finally, the wells were washed three times with Buffer A, and 100 µL peroxidase substrate TMB was added, and the reaction was terminated after 30 min with 50 µL of 450 nm of stop solution for TMB. The absorbance was determined at 450 nm with a Microplate Reader (Bio-Rad, Hercules, CA, USA). The best-fit 50% inhibitory concentration (IC_50_) values for the different compounds were calculated by fitting the data with nonlinear regression using GraphPad Prism (GraphPad, San Diego, CA, USA).

### 2.2. Cell Culture

The human glioblastoma U87-luc and primary GBM cells were obtained from ATCC (Manassas, PA, USA) and a generous gift from University of Pittsburgh Medical Center (Pittsburgh, PA, USA) and were grown in Dulbecco’s Modified Eagle’s Medium (DMEM) supplemented with 10% fetal bovine serum, 10% penicillin, and 1% streptomycin. The cells were cultured at 37 °C to sub-confluence and treated with 0.25% (*w*/*v*) trypsin/ethylenediaminetetraacetic acid (EDTA) to induce cell release from the flask. The cells were washed with a culture medium that was free of phenol red and fetal bovine serum, and then counted.

### 2.3. Cell Proliferation Assay

The glioblastoma cells (U87-luc) and primary cells GBM 101813, GBM 021,913 were seeded in 96-well plates (0.5 million cells per well) and treated with Compounds **1**, **2**, and **3** at 5 concentrations (1, 3, 10, 30, and 100 µM). At the end of the experiments, the cell cultures were supplemented with MTT reagent (3-(4,5-dimethylthiazol-2-yl)-2,5-diphenyltetrazolium bromide) and incubated for an additional 4 h. Then, dimethyl sulfoxide (0.1% DMSO) was added to the cell culture to dissolve the formazan crystals and incubated for 10 min at room temperature. The absorbance rate of the cell cultures was read at 570 nm by using a Microplate Reader. All the reactions were performed in triplicate. The measured data of the cellular proliferation were calculated using the viability values of the untreated control cells (100%).

### 2.4. Chorioallantoic Membrane Assay (CAM) 

Neovascularization was examined in the CAM model, as previously described [18,19,20,21]. We purchased 10-day-old chick embryos purchased from Charles River Avian Vaccine Services (Norwich, CT, USA) and incubated them at 37 °C with 55% relative humidity. A hypodermic needle was used to make a small hole in the shells at the air sacs, and a second hole was made on the broadside of the eggs, directly over an avascular portion of the embryonic membrane that was identified by candling. A false air sac was created beneath the second hole by the application of negative pressure at the first hole, causing the CAM to separate the shell. A window of approximately 1.0 cm^2^ was cut in the shell over the dropped CAM using a small craft grinding wheel (Dermal, Division of Emerson Electric Co. Racine, WI, USA), allowing for direct access to the underlying membrane. b-FGF (10 ng/CAM) was used as a standard proangiogenic agent, and sterile disks of No. 1 filter paper (Whatman International, Kent, UK) were pretreated with 1 µg/CAM of Compounds **1**, **2**, and **3**, air-dried under sterile conditions and placed on the CAMs. 

### 2.5. Microscopic Analysis of CAM Sections

After incubation at 37 °C with 55% relative humidity for 3 days, the CAM tissue directly beneath each filter disk was resected from each CAM sample. The tissues were washed three times with PBS, placed in 35 mm Petri dishes (Nalge Nunc, Rochester, NY, USA), and examined under SV6 stereomicroscope (Carl Zeiss, Thornwood, NY, USA) at ×50 magnification. Digital images of the CAM sections exposed to the treatment filters were collected using a 3-CCD color video camera system (Toshiba America, New York, NY, USA), and analyzed with Image-Pro software (Media Cybernetics, Silver Spring, MD, USA). The number of vessel branch points contained in a circular region equal to the area of each filter disk were counted. There was 1 image counted in each CAM preparation, and findings from 8 CAM preparations per each treatment condition. The results are presented as the mean ± SD of new branch points in the collected samples from each treatment condition.

### 2.6. Animals

Immunodeficient female NCr nude homozygous mice aged 5–6 weeks and weighing 20–25 g were purchased from Taconic Biosciences, Inc (Germantown, NY, USA). All animal studies were conducted at the animal facility of the Veteran Affairs Medical Center (Albany, NY, USA) in accordance with the approved institutional guidelines for humane animal treatment and according to the current guidelines. The mice were kept under specific pathogen-free conditions and housed under controlled conditions of temperature (20–24 °C) and humidity (60–70%) and a 12 h light/dark cycle with ad libitum access to water and food. The mice were allowed to acclimatize for 5 days before the study.

### 2.7. Glioblastoma Xenografts

For the subcutaneous (s.c.) glioma tumor model, the study was conducted as diagrammed in Figure 2. U87-luc cells were harvested, suspended in 100 μL of DMEM with 50% Matrigel^®^ (Pasadena, TX, USA) and 2 × 10^6^ cells were implanted s.c. dorsally in each flank to achieve two independent tumors per animal. Immediately prior to the initiation of treatments, the animals were randomized into treatment groups (5 animals/group) by tumor volume measurements with Vernier calipers. Treatments began after the detection of a palpable tumor mass (4–5 days post-implantation). Because these compounds had different percentages of the active tetrac portion (s) of the molecule relative to the full molecule, we dosed the compounds at equivalent moles/kg triazole tetrac (TAT) levels rather than mg/kg of the intact compound. Thus, compounds were dosed at 0.354 µmol/kg, 1.06 µmol/kg, and 3.54 µmol/kg TAT. The treatments were the control (PBS), Compound **1** (0.354, 1.06, 3.54 mg/kg), Compound **2** (0.354, 1.06, 3.54 mg/kg), and Compound **3** (0.354, 1.06, 3.54 mg/kg). The agents were administered daily, s.c., for 21 days (ON Treatment), and in another set of animals, the compounds were administrated daily for 21 days, followed by 21 days of discontinuation (ON Treatment + OFF Treatment). The animals were then humanely sacrificed, and the tumors were harvested. The tumor weights and the cell viabilities (bioluminescent signal intensity) were measured.

### 2.8. Tumor Volume and Weight

The tumor widths and lengths were measured with calipers at 3-day intervals during the ON and ON + OFF studies, and the volumes were calculated using the standard formula W × L^2^/2. The tumor weights measured were of harvested lesions following animal sacrifice.

### 2.9. Bioluminescence

The mice were injected s.c. with 50 μL D-luciferin (30 mg/mL). They were anesthetized using isoflurane, and post-luciferin administration mice were imaged in an in vivo imaging system (Xenogen-IVIS spectrum, PerkinElmer Inc., Waltham, MA, USA). Photographic and luminescence images were taken at a constant exposure time. Xenogen IVIS Living Image software (version 3.2) was used to quantify non-saturated bioluminescence in regions of interest (ROI). Bioluminescence was quantified as photons/s for each ROI. Ex vivo tumor imaging was performed to confirm the signal intensity in the tumors after the termination of the study. 

### 2.10. Histopathology

The tumors were fixed in 10% formalin, placed in cassettes, and dehydrated using an automated tissue processor. The processed tissues were embedded in paraffin wax and the blocks were trimmed and sectioned to about a 5 × 5 × 4 µm size using a microtome. The tissue sections were mounted on glass slides using a hot plate and subsequently treated in the order of 100%, 90%, and 70% ethanol for 2 min. Finally, the tissue sections were rinsed with water, stained with Harris’s hematoxylin and eosin (H&E), and examined under a light microscope.

### 2.11. Statistical Analysis

Statistical analysis was performed with GraphPad Prism 7 software. Data are presented as the mean ± SD. For comparison between two or more sets of data, ANOVA was used. * *p* < 0.05, ** *p* < 0.01, and *** *p* < 0.001 were considered statistically significant.

## 3. Results 

### 3.1. Binding Affinity of Compounds to Integrins

To evaluate the specificity and selectivity of TATs to integrins, we investigated for the subtypes αvβ1, αvβ3, αvβ5, αvβ6, IIbβ3, α5β1, and αvβ3 in an integrin–ligand binding assay. The lowest IC_50_ values of Compounds **1**, **2**, and **3** were 0.14, 0.23, and 0.36 nM, respectively, were observed for αvβ3 (Figure 3). No significant changes in IC_50_ values were observed for Compounds **2** and **3** when compared to Compound **1**. 

Integrins are adhesion receptors that play an essential role in cell–cell communications. αvβ3 is an attractive target for therapeutic intervention because of its presence in many types of cancer cells and their neovasculature, which plays a key role in tumor growth, tumor angiogenesis, and metastasis. 

### 3.2. Effect of TATs on Cell Proliferation of U87-Luc Cells

To compare the in vitro anticancer activity of the three TATs, an MTT assay was used. As shown in Figure 4, we evaluated the effects of these compounds on the growth of human glioblastoma U87-luc cell lines and primary cells (GBM 101813, GBM 021913). In the MTT assay, the U87-luc cell line showed decreases in proliferation of 56%, 59%, and 58% at 24 h, and 42%, 44%, and 43% at 48 h, with 100 μM of Compounds **1**, **2**, and **3**, respectively compared to the untreated cells (Figure 4C,D). For the GBM 101813, cells with 100 μM of Compounds **1**, **2**, and **3** showed decreases in proliferation of 52%, 54%, and 55% at 24 h, and 41%, 43%, and 45% at 48 h, respectively (Figure 4C,D). Further, GBM 021913 showed decreases in cell proliferation of 54%, 57%, and 57% at 24 h, and 48%, 52%, and 50% with 100 μM of Compounds **1**, **2**, and **3** compared to the untreated cells (Figure 4E,F). 

### 3.3. Anti-Angiogenesis Efficacy of TATs 

To compare the anti-angiogenic efficacy of the three TATs, a CAM assay was used. As shown in Figure 5, a basic fibroblast growth factor (FGF2 or b-FGF) was used to stimulate angiogenesis, and then the compounds were administrated. Compounds **1**, **2**, and **3** showed maximum inhibition of the number of vessel branch points (angiogenesis) at 1 µg/CAM. No statistically significant changes in the percentages of inhibition of angiogenesis were observed between the three TATs. The TAT molecules also showed maximum inhibition of angiogenesis in the presence of different growth factors (VEGF, HGF, and in combination).

### 3.4. Antitumor Effect 

With the intent to study the in vivo antitumor efficacies of Compounds **1**, **2**, and **3** on tumor growth, U87-luc glioblastoma cells were implanted in each flank of the animals, and then the mice were treated daily for 21 days with Compounds **1**, **2**, and **3**. The tumor volumes significantly decreased when treated with Compounds **1**, **2**, and **3** at 0.354, 1.06, and 3.54 µmole/kg, respectively, compared to the controls (Figure 6). All the treatments at 0.354, 1.06, and 3.54 µmole/kg significantly reduced the tumor weight after daily treatment for 21 days. The xenograft weights and tumor cell viabilities decreased by >90% with all doses (ON Treatment, *** *p* < 0.001) compared to the control (Figure 7A). In the second group, Compound **1**-treated mice, the xenografts were observed for an additional 21 days with no further treatment (ON Treatment + OFF Treatment). There was no re-growth of tumors in these groups of animals and the absence of cell viability persisted (Figure 7B). Similar results were obtained from mice treated daily with Compounds **2** and **3** for 21 days (ON Treatment) and another group treated daily for 21 days followed by discontinuation for 21 days (ON + OFF Treatment).

The in vivo luminescent signals of viable cancer cells were quantified (photons/second) for the different groups using a Xenogen-IVIS Spectrum. A statistically significant (*p* < 0.001) decrease of viable U87-Luc cells was observed in groups treated with TATs compared to the control. No significant differences were observed when comparing the treated groups (Figure 7C,D). 

Further, the histological sections obtained from the U87 xenografts were used to evaluate the antagonist treatments on cell proliferation. A large necrotic area was observed in the tumor masses from all doses of the treatment groups. However, there was no significant difference between the three antagonist treatments (Figure 8).

### 3.5. Transthyretin (TTR) Binding Assay

Further, we tested the ability of TTR binding using competitive fluorescence binding assay. FITC-T_4_ and TTR were mixed in a 96-well plate and incubated with different concentrations of Compounds **1**, **2**, and **3**, and the intensity of fluorescence was measured at 518 nm. The IC_50_ values of Compounds **1**, **2**, and **3** were 5.5 nm, 5.6 nm, and 4.8 nm, respectively (Figure 9). 

## 4. Discussion

The integrin αvβ3 plays a critical role in glioblastoma-associated biological processes, making it an important target for the development of novel targeted ligands. GBM is a thyroid hormone-dependent tumor, and this effect was mediated via non-genomic actions of the cell-surface receptor on integrin αvβ3 [22]. Although various integrin ligands have been reported, most of them are universal ligands for multiple integrin receptors and show a limited binding affinity for integrin αvβ3. A number of in vitro and in vivo studies have supported the role of thyroid hormones (L-thyroxine, T4; 3,5,3′-triido-L-thyronine, T3) in the proliferation of tumor cells. In the present study, we compared the therapeutic efficacy of the two integrin αvβ3 antagonists, the monomer P-m-TAT (Compound **3**) and P-bi-TAT dimer, (Compound **2**) with P-bi-TAT dimer (Compound **1**). Recently, we showed that the incorporation of a triazole group and PEG molecules within P-bi-TAT (Compound **1**), and without any change to the carboxylic acid group, significantly increased the integrin binding affinity compared to the tetrac [11]. Our group previously compared the potency of NDAT in in vitro and in vivo studies using U87 glioblastoma cells [12]. The chain length of PEG that restricts the nuclear translation of the thyromimetic tetrac within the molecule as well the improved solubility in an aqueous buffer for subcutaneous injection has to be greater than 1200 Dalton, which is why we used PEGs between 1600–4000 Daltons [5,11].

In the past decade, our studies have shown the αvβ3-dependent antiproliferative, anti-angiogenic, and anticancer properties of agonist thyroid hormones (T4, T3) by tetrac in various cancer types. In the present study, the inhibition of U87 cell growth by TATs was comparable at a higher drug concentration (100 µM), but there was increased sensitivity to P-bi-TAT (Compound **1**) at a lower drug concentration of the used agents. Cody et al., 2007 showed that unmodified tetrac may penetrate cells and can interact with the thyroid hormone nuclear receptor to where it is a low potency agonist (thyromimetic) [23]. On the other hand, P-bi-TAT (Compound **1**) does not gain access to the cell nucleus and shows a more robust antiproliferative effect. It has been well documented that increasing PEG substitution can lower the binding affinities of different therapeutics [24,25,26,27].

In earlier in vitro studies, we showed that three rodent glioma cell lines proliferated in response to thyroid hormone, which is blocked by tetrac [11]. Beyond antiproliferation at the level of the tumor cell, a second important facet of the properties of αvβ3 antagonists is that they have anticancer efficacy by multiple mechanisms. Here, the in vivo antitumor efficacies of the αvβ3 antagonists were evaluated in U87-luc glioblastoma tumor-bearing nude mice, and the compounds significantly reduced tumor volumes and impaired tumor growth in a dose-dependent manner by suppressing angiogenesis (ON Treatment). In the second group of treated mice, the xenografts were observed for an additional 21 days with no further treatment (ON + OFF Treatment). No regrowth of tumors was observed, and the absence of cell viability persisted. One explanation for these observed effects is that tetrac impairs tumor growth by blocking angiogenesis and by impairing the endothelial cell function rather than by impeding tumor cell growth directly. We have ascribed conventional pro-apoptotic activity to tetrac that would account for the progressive decrease in tumor volume that occurred over 21 days of treatment.

Previously, our group formulated a polymeric nanoparticle, NDAT, against a variety of xenografts. Chemical changes to the tetrac molecule at the outer ring hydroxyl by adding a triazole and PEG molecule did not allow the agent to gain access to the cell interior and thus, the tetrac that is ether-bonded to the PLGA particle via the outer ring hydroxyl can act only at the integrin receptor, where it is exclusively an antagonist and not at the nuclear receptor for thyroid hormone. Further, the histopathological sections represent that the extensive necrosis induced in the tumor mass is present in all treated tumors, causing apoptosis.

The following are limitations of the study: GBM tumor implants were xenografted versus orthotopically implanted in the brain to allow for an extended investigation of the effect of TAT treatment for up to 3 weeks in one group, and in another group, the TAT treatment for up to 3 weeks was followed by 3 weeks off treatment to examine the impact on tumor re-growth or relapse. A total of 6 weeks (3 weeks ON treatment + 3 weeks OFF) was the maximum duration that the implanted animals had minimal pain and distress, and significant pain and distress developed beyond that duration.

We have also developed satisfactory evidence that TATs cross the blood–brain barrier. The luminescent signals of the single molecular target on αvβ3, the target that, when activated by chemically modified tetrac, regulates a network of intracellular signaling pathways and plasma membrane functions, and further, controls specific gene transcription and cell surface vascular growth factor receptor functions that are highly relevant to cancer and cancer-linked angiogenesis. Previous studies showed that αvβ3 antagonists’ multivalency results in increased binding affinity, which then improved targeted therapeutic delivery [11,28,29]. However, despite many studies over years, there are no reports that have demonstrated improved therapeutic effectiveness of dimer αvβ3 antagonists over monomer αvβ3 antagonists.

The CENTRIC phase 3 trial, a multicenter, randomized, open-label, phase 3 trial that assessed cilengitide in addition to the standard of care treatment against newly diagnosed GBM, which failed to improve survival [30]. Therefore, the role of integrins as a target for glioblastoma can be debated. The failure of cilengitide, as pointed out above, is mainly due to the kinetics and the fact that cilengitide acts as a partial agonist; αvβ3 integrin is activated when cilengitide concentration declines because of its fast off-rate from the αvβ3 integrin and its stability and short half-life [31]. In contrast, our TAT derivatives are pure antagonists, stable along with a fast on-rate and a slow off-rate of binding to the αvβ3 integrin.

## 5. Conclusions

In conclusion, we found that the three TATs integrin αvβ3 antagonists showed no significant differences among them in their binding affinities to the αvβ3 receptor. Furthermore, the biological studies showed that decreasing PEG linker sizes and mono-TAT versus bi-TAT molecules resulted in no significant change in antitumor efficacy against glioblastoma.

## Figures and Tables

**Figure 1:** Schematic structures of (**A**) P_4000_-bi-TAT (Compound **1**), (**B**) P_1600_-bi-TAT (Compound **2**), and (**C**) P_1600_-m-TAT (Compound **3**). In the structure, ‘n’ and ‘m’ indicate the PEG size. (**A**,**B**) differ in PEG size, with a molecular weight of 4000 (n ~ 90) and 1600 (n = 35), respectively.

**Figure 2:** Protocol for subcutaneous administration of compounds in mice with U87-luc xenografts. (**A**) ON Treatment: the compounds were administered daily, s.c. for 21 days, and (**B**) ON + OFF Treatment: the compounds were administrated daily for 21 days followed by 21 days of discontinuation. At the end of the study, the animals were humanely sacrificed, and the tumors were harvested.

**Figure 3:** Binding affinity of TATs for the integrins αvβ1, αvβ3, αvβ5, αvβ6, IIbβ3, α5β1, and αvβ3. (**A**) Compound **1**, (**B**) Compound **2**, (**C**) Compound **3**. Dose-response curve (mean IC_50_ (nM) ± SD) of three independent experiments. *x*-axis show Log Concentrations from −12 to −6.

**Figure 4:** Cell proliferation assay. U87-luc and primary (GBM 101813, GBM 021913) cells were incubated with Compounds **1**, **2**, and **3** at different concentrations (1, 3, 10, 30, and 100 µM) for 24 h and 48 h and were measured with MTT assay. (**A**,**B**) U87-luc; (**C**,**D**) GBM 101813; (**E**,**F**) GBM 021913. Values are presented as the mean ± S.D of three independent experiments. *** *p* < 0.001, ** *p* < 0.01, * *p* < 0.05 compared to the control (PBS).

**Figure 5:** Inhibition of angiogenesis in chick chorioallantoic membrane (CAM). With the development of small new blood vessels, typical neovascularization was visible with CAM assay. (**A**) Images represent the inhibition of the b-FGF (10 ng/CAM)-induced angiogenesis by Compounds **1**, **2**, and **3** at 1 µg/CAM. (**B**) Data illustrate the decrease of compounds. Values are presented as the mean ± S.D *** *p* < 0.001, compared to the control.

**Figure 6:** Anti-cancer effects of Compounds **1**, **2**, and **3** on tumor volumes. (**A**) Compound **1**; (**B**) Compound **2**; (**C**) Compound **3**. U87-luc glioblastoma cells implanted mice were treated daily with Compounds **1**, **2**, and **3** (ON Treatment) for 21 days, and in the second group, the xenografts were observed for an additional 21 days with no further treatment (ON Treatment + OFF Treatment). Values are presented as the mean tumor volume (mm^3^) ± S.D. *** *p* < 0.001, ** *p* < 0.01, * *p* < 0.05, compared to the control.

**Figure 7:** Antitumor effects of Compounds **1**, **2**, and **3** on xenografts. (**A**,**B**) Tumor weight; (**C**,**D**) luminescence signals in xenografts; (**E**) representative IVIS images of luminescent signals in tumors. Values are presented as the mean ± S.D.

**Figure 8:** Histopathological images of H&E staining of glioblastoma xenografts in nude mice treated with Compounds **1**, **2**, and **3**. The scale bar is 10×. Complete infiltration with the malignant cells ~100% was observed in the controls. In the treatment groups, necrosis, and hyalinization > 90% were observed.

**Figure 9:** TTR binding assay. TTR and FITC-T_4_ were mixed and incubated with different concentrations of Compounds **1**, **2**, and **3**. Competitive fluorescence binding curves (mean IC_50_ ± SD) of three independent experiments. *x*-axis shows Log Concentrations from −11 to −5.

## Data Availability

The data presented in this study are available on request from the corresponding author.
